This article has been retracted.

# M3 muscarinic acetylcholine receptors regulate epithelial–mesenchymal transition, perineural invasion, and migration/metastasis in cholangiocarcinoma through the AKT pathway

**DOI:** 10.1186/s12935-018-0667-z

**Published:** 2018-11-06

**Authors:** Yujie Feng, Xiao Hu, Guangwei Liu, Lianfang Lu, Wei Zhao, Fangzhen Shen, Kai Ma, Chuandong Sun, Chengzhan Zhu, Bingyuan Zhang

**Affiliations:** 1 Department of Hepatobiliary and Pancreatic Surgery, The Affiliated Hospital of Qingdao University, No. 16 Jiangsu Road, Qingdao, 266003 Shandong China; 2 Department of Outpatient, The Affiliated Hospital of Qingdao University, No. 16 Jiangsu Road, Qingdao, 266003 Shandong China; 3 Department of Oncology, The Affiliated Hospital of Qingdao University, No. 16 Jiangsu Road, Qingdao, 266003 Shandong China

**Keywords:** Cholangiocarcinoma, M3 muscarinic acetylcholine receptors, Perineural invasion, Epithelial–mesenchymal transition, AKT

## Abstract

**Background:**

Cholangiocarcinoma is a highly malignant tumor type that is not sensitive to radiotherapy or chemotherapy due to aggressive perineural invasion and metastasis. Unfortunately, the mechanisms underlying these processes and the signaling factors involved are largely unknown. In this study, we analyzed the role of M3 muscarinic acetylcholine receptors (M3-mAChR) in cell migration, perineural invasion, and metastasis during cholangiocarcinoma.

**Methods:**

We assessed 60 human cholangiocarcinoma tissue samples and 30 normal biliary tissues. Immunohistochemical staining was used to detect M3-mAChR expression and the relationship between expression and clinical prognosis was evaluated. The biological functions of M3-mAChR in cholangiocarcinoma cell migration, perineural invasion, and epithelial–mesenchymal transition (EMT) were investigated using the human cholangiocarcinoma cell lines FRH0201 and RBE in conjunction with various techniques, including agonist/antagonist treatment, RNA interference, M3-mAChR overexpression, dorsal root ganglion co-culturing, immunohistochemistry, western blotting, etc.

**Results:**

M3-mAChR were highly expressed in cholangiocarcinoma tissue and expression was closely related to differentiation and lymphatic metastasis, affecting patient survival. Treatment with the M3-mAChR agonist pilocarpine and M3-mAChR overexpression significantly promoted migration and perineural invasion, while the M3-mAChR antagonist atropine blocked these effects. Similarly, M3-mAChR knock-down also weakened cell migration and perineural invasion. The expression of phosphatase and tensin homolog, AKT, E-cadherin, vimentin, and Snail, which are components of the phosphatidylinositol 3-kinase/AKT signaling pathway and EMT, were altered by pilocarpine, and these effects were again blocked by atropine. Notably, AKT knock-down decreased M3-mAChR expression and reversed the downstream effects of this receptor.

**Conclusions:**

M3-mAChR are involved in tumor cell migration, perineural invasion, and EMT during cholangiocarcinoma, and these effects are modulated via the AKT signaling pathway.

## Background

Cholangiocarcinoma, which originates from biliary epithelial cells, is a type of malignant tumor that is characterized by low diagnostic rates and high fatality rates [1]. Concealed pathogenesis, lack of early diagnostic markers, and low sensitivity to conventional radiotherapy and chemotherapy treatments are the crucial reasons underlying the poor prognosis of cholangiocarcinoma patients. Currently, surgical resection is the only effective treatment method for this disease. Moreover, recent studies have found that perineural invasion is a common biological characteristic of cholangiocarcinoma and is closely related to postoperative recurrence rates and prognoses [2].

Cholangiocarcinoma undergoes perineural invasion early in development and involves tumor cells surrounding the nerve fibers, entering the perineurium, and spreading via local infiltration and metastasis. Recent studies have shown that the biliary system is rich in autonomic nerves, and biliary tract malignancy occurs near the celiac plexus; thus, tumor cells are more likely to invade the surrounding nerve plexus, causing perineural invasion [3]. Another study reconstructed the perineural invasion and metastasis processes that occur during cholangiocarcinoma by computer-assisted three-dimensional (3D) analysis and formed 3D images of cholangiocarcinoma to display existing small vessels, lymph vessels, and nerve fibers around the tumor [4]. They concluded that tumor cells survive independently in spaces around the nerves, including in the small vessels and small lymph vessels. Accordingly, perineural invasion was found to be the fifth self-existent route of metastasis following direct invasion and metastasis, implantation metastasis, lymphatic metastasis, and blood metastasis of abdominal tumors. Metastasis occurs in the nerve fibers via jumping, meaning that cholangiocarcinoma can either invade and metastasize to the liver through the perineural space or metastasize to the retroperitoneal ganglions. This is also why cholangiocarcinoma is difficult to cure.

As an important digestive organ, the biliary system regulates biliary secretion and excretion and is surrounded by vagus nerves, which can interact with the liver vascular system and inevitably affect the pathophysiology of the biliary epithelium [5]. However, while these systems interact and affect the health and function of each other, for the cancer cells to spread from the primary site, they must develop migratory and invasive properties. Epithelial-to-mesenchymal transition (EMT) is a phenomenon in which epithelial cells lose their original polarity and transform into Leydig cells. EMT is comprised of a series of intricate biological and biochemical changes that cause the cell to lose its differentiated epithelial-like state and gain a more mesenchymal-like phenotype. Moreover, the EMT is closely related to tumorigenesis, local invasion, distant metastasis, and tumor resistance [6–9] and appears to play a distinct role in cholangiocarcinoma [10]. The various processes involved in cholangiocarcinoma, including perineural invasion, metastasis, and EMT, likely require complex signaling pathway function as well as a host of independent factors, many of which have not been elucidated.

Muscarinic acetylcholine receptors (mAChRs) are members of the G protein-coupled receptor family and include five receptor subtypes (M1, M2, M3, M4, and M5) [11]. The M3-mAChR are mainly distributed in the digestive tract glands and vascular smooth muscles and modulate glandular secretion and smooth muscle relaxation. Various studies have also shown that M3-mAChR play an important role in the proliferation and invasion of cancer cells [12–14]. However, the role of M3-mAChR in cholangiocarcinoma has not been evaluated.

In this study, we investigated the function of M3-mAChR during perineural invasion, metastasis, and EMT in cholangiocarcinoma. To our knowledge, this is the first time M3-mAChR-mediated regulation has been explored in cholangiocarcinoma.

## Methods

### Patients and tissue specimens

We collected paraffin-embedded biliary pathology tissues obtained during surgical resection at the Affiliated Hospital of Qingdao University from December 2008 to December 2013. The samples included 60 cholangiocarcinoma tissues and 30 normal biliary tissues (from patients with choledochocysts and liver transplantation). Patient data was also collected. None of the patients had undergone radiotherapy or chemotherapy/drugs treatment before the operation. All procedures in this study that involved human participants were performed in accordance with the 1964 Helsinki declaration and its later amendments. The protocol was approved by the Ethics Committee of The Affiliated Hospital of Qingdao University. Informed consent was obtained from all individual participants included in the study.

### Immunohistochemistry

The paraffin-embedded biopsy tissue specimens were cut into 4-μm-thick sections and deparaffinized. The sections were pretreated and incubated with primary anti-M3 mAchR antibodies (1:1000; Abcam, Cambridge, UK) overnight at 4 °C according to the manufacturer’s instructions. Then, the sections were incubated with secondary antibodies for 30 min, stained with diaminobenzidine, and finally, counterstained with hematoxylin. The stained sections were then imaged (400×; OLYMPUS, Tokyo, Japan). Positive staining in the basement membrane was manifested as a brownish-yellow color.

For statistical analysis, 10 random fields of the tumor were selected in each section, and 100 cells from each field were counted. The samples were then graded according to the proportion of positive cells to the total number of cells. When the percentage of positively stained cholangiocarcinoma cells was less than 25%, the result was considered negative. Alternatively, when the percentage was between 25 and 55% or more than 55%, the staining was described as positive and strongly positive, respectively.

### Cell lines, culture conditions and reagents

The cholangiocarcinoma cell lines FRH0201 and RBE were purchased from the Shanghai Cell Bank of the Chinese Academy of Sciences. The cell lines were all authenticated. The cells were grown and cultivated in RPMI-1640 medium supplemented with 10% newborn calf serum (Thermo Scientific Hyclone, USA) in an incubator containing 5% CO_2_ at 37 °C. M3-mAChR agonist pilocarpine and M3-mAChR antagonist atropine were purchased from Sigma-Aldrich (Taufkirchen, Germany).

### Constructing the lentivirus vector for RNAi and receptor overexpression

The most effective M3-targeting small hairpin RNA (shRNA) sequences (5′-GCAGTGACAGTTGGAACAACA-3′) were transfected into the cultured cells using Lipofectamine 2000 Reagent (Invitrogen, Carlsbad, CA, USA). M3-NC (5′-TTCTCCGAACGTGTCACGT-3′) was used to generate the negative (scrambled) control lentiviral vectors. Lentivirus was added to the cells according to the manufacturer’s recommended protocol.

The high-copy plasmid pcDNA 3 1(+) (Invitrogen, Carlsbad, CA, USA) harbouring the complete cDNA of the human mAchR3 was performed according to the manufacturer’s protocol using a commercially available kit (Qiagen, Hilden, Germany).

### RNAi treatment

FRH0201-M3 cells were transfected with siAKT (5′-TTGTACGCAGAGAGAATAACT-3′), using the Lipofectamine transfection reagent (Invitrogen) for 48 h. Retrovirus packaging and transfection were conducted according to the manufacturer’s instructions.

### Quantitative real-time polymerase chain reaction (qRT-PCR)

Total RNA was extracted from cultured cells using TRIzol reagent in a one-step method according to the manufacturer’s instructions. Primer design was performed using Primer5 software with sequences for human M3-mAChR obtained from GenBank. The following primers were used in this study:M3-mAChR (forward, 5*′*-CACAATAACAGTACAACCTCGCC-3*′* and reverse, 5*′*-GCCAGGATGCCCGTTAAGAAA-3*′*). internal control GAPDH (forward, 5*′*-GCACCGTCAAGGCTGAGAAC-3*′* and reverse, 5*′*-TGGTGAAGACGCCAGTGGAT-3*′*. M3-mAChR gene expression was quantitated using the 2^−∆∆Ct^ method. The data are presented as the fold change compared to the specified controls using an average result of three independent experiments. Differences were considered biologically relevant when the fold change was > 2.0 or < 0.5 [15].

### Western blot analysis

Whole cell lysates were prepared using RIPA lysis buffer and protease inhibitor (keyGEN, Nanjing, China), and the protein concentrations were determined using a BCA kit (Thermo Scientific™). A total of 50 μg of protein was loaded into each well of a sodium dodecyl sulfate polyacrylamide gel electrophoresis (SDS-PAGE) gel, and the proteins were separated. After the proteins were transferred to a polyvinylidene difluoride membrane, the membranes were blocked with 5% nonfat dried milk for 2 h. Next, the membranes were incubated overnight with primary antibodies targeting M3-mAChR, phosphatase and tensin homolog (PTEN), AKT, E-cadherin, vimentin, and Snail (all purchased from Santa Cruz Biotechnology, Santa Cruz, CA, USA) at 4 °C. The membranes were then incubated with secondary antibodies for 2 h at room temperature. Finally, the protein bands were visualized using enhanced chemiluminescence, and their intensity was quantified.

### Migration assay

For the transwell migration assays, 10^5^ cells were seeded in 100 μL of serum-free Dulbecco’s modified Eagle’s medium in fibronectin-coated polycarbonate membrane inserts in a transwell apparatus. The diameter of the membrane micropores was 8 μm. A total of 600 μL of RPMI-1640 culture medium with 10% serum was added to the lower wells. After culturing cells for 36 h at 37 °C, the transwell chambers were removed and washed with phosphate-buffered saline three times. Cells that had not invaded were removed using aseptic cotton buds, and the chambers were then fixed in 4% formalin solution for 20 min. Next, cells on the chambers were stained with 0.1% crystal violet for 15 min and then imaged under an optical microscope. Cells in 10 fields were counted (400× magnification). The experiment was performed in triplicate.

### Dorsal root ganglion isolation and ex vivo culture

As described in a previous study [16], newborn Kunming mice (24 h old) were disinfected using 75% ethyl alcohol, sacrificed by cervical dislocation, and fixed in the prone position. The mediodorsal skin was cut using sterile eye scissors to expose the muscles of the back. Taper eye scissors were then used to cut an opening and expose the spinal cord, which was excised and washed with normal saline several times, until the dorsal root ganglion (DRG) could be observed. Next, the DRG was carefully removed using smooth microforceps and washed once in normal saline. The washed DRG was then transferred into a 24-well plate, and thawed Matrigel (BD Biosciences, Franklin Lake, NJ, USA) was added to completely cover it. The Matrigel-coated DRG was then incubated at 37 °C for 30 min until coagulation. Notably, all of these procedures involving the care and use of laboratory animals were performed in accordance with the principles and standards set forth in the Principles for Use of Animals (National Guide for Grants and Contracts).

### DRG immunohistochemical staining

#### Nissl staining to observe the state of nerve cell viability

Remove the neurons from which the culture solution was discarded, and wash it with 0.01 mol/L PBS three times for 5 min each time. Then 4% paraformaldehyde was fixed at room temperature for 1 h, and washed with 0.01 mol/L PBS for 3 times for 5 min each time followed by 0.1% toluidine blue dyeing at 37 °C for 10 min. After the final 95% ethanol separation, the cells were dehydrated in 50%–100% gradient ethanol for 3–5 min each time. The xylene was transparent and the gel was sealed, and then the neuron viability was observed under a microscope.

#### Neurofilament protein (NF) immunocytochemical staining of DRG

Co-infiltrate and purify the cultured DRG, discard the culture solution and wash it with 0.0 l mol/L PBS for 3 times for 5 min each time; 4% paraformaldehyde was fixed at room temperature for 1 h, washed with PBS; 0.3% H_2_O_2_ methanol was added., placed for 10 min to remove endogenous catalase, washed with PBS and moved to a wet box. Add 10% sheep serum to the coverslip, add 3 drops per well, and incubate in a 37 °C oven for 30 min; after aspirating the blocking solution, l:200 rabbit anti-mouse NF antibody (Beyotime, Shanghai, China) 3 drops per tablet, at 4 °C refrigerator save. Immediately after the PBS cleaning, add goat anti-rabbit IgG (1:200 biotinylated, Beyotime, Shanghai, China) on the coverslip, 3 drops per well, incubate in a 37 °C oven, and wash with PBS after 30 min. Add the ready-to-use ABC solution onto the coverslip and incubate in a 37 °C oven for 30 min; wash with PBS, add DAB coloring solution for 8–10 min, then rinse again with PBS. Finally, dehydrated in 50% concentration gradient ethanol, about 5 min each time, xylene was transparent and the gel was sealed, and then the axon extension of each group was observed under a microscope.

### Co-culturing of DRG segments and RBE cells

For co-culturing, untreated RBE cells in the logarithmic growth phase were added to each well of the 24-well plate containing a Matrigel-coated DRG at a concentration of 2.5 × 10^4^ cells/well in 500 μL of medium (RPMI-1640 containing serum). The DRGs were treated as follows: MOCK (medium + RBE cells), ShM3 (medium + ShM3-treated RBE cells), PILO [medium + RBE cells + pilocarpine (1.0 mM)]; ATR [medium + RBE cells + atropine (0.1 mM)], and PILO + ATR [medium + RBE cells + pilocarpine (1.0 mM) + atropine (0.1 mM)]. Cell adhesion to the DRG nerve fibers was observed using an inverted microscope every 4 h. After 72 h, the number of cholangiocarcinoma cells adhering to nerve fibers was quantified.

### General matrix metalloproteinase (MMP) activity assay

The general activity of MMP enzymes was determined using an assay kit (ab112146, Abcam, Cambridge, MA, USA) according to the manufacturer’s protocol. In brief, experimental cells were seeded into triplicate wells of 6-well plates and allowed to attach overnight, then starved with serum free media for another 18 h. A kinetic measurement was then performed for the MMP activity by taking medium samples at 5 min intervals over a 1 h period after starting the reaction by using a microplate reader with a filter set of Ex/Em = 490/525 nm.

### Statistical analysis

Statistical analyses were performed using SPSS 17.0 software. Each value in the present study was obtained from at least three independent experiments. Data are presented as the mean ± standard error of the mean (SEM). Survival analyses and cumulative recurrence rates were assessed using the Kaplan–Meier method and the log-rank test. The difference between two groups was evaluated with the Student’s *t*-test and was considered statistically significant when *P* < 0.05.

## Results

### Clinicopathological features and patient demographics

All of the cases of cholangiocarcinoma (n = 60; 43 men, 17 women; median age, 56 years; range, 30–82 years) were diagnosed as adenocarcinoma. Of these, 46 cases (76.67%) had lymphatic metastasis, while 14 (23.33%) did not. A total of 18 cases (30%) of high differentiation and 42 cases (70%) of moderate or low differentiation were observed. Furthermore, after classification the tumors according to the Union International Control Cancer TNM staging system [17], 16 cases (26.67%) were found to be stage I-II, while 44 cases (73.33%) were stage III-IV. Finally, we found that 53 cases (88.33%) of them had perineural invasion and the remaining 7 cases (11.67%) without perineural invasion.

### M3-mAChR is highly expressed in cholangiocarcinoma and plays an important role in metastasis and prognosis in cholangiocarcinoma patients

Using immunohistochemistry, we observed M3-mAChR to be highly expressed in histopathological sections from cholangiocarcinoma tissues, but was found at lower levels in normal biliary tissues, with positive rates of 90% (54/60) and 3.33% (1/30), respectively (*P* < 0.01; Fig. 1a, b). In the positive tissues, M3-mAChR expression was mainly distributed in granules or sheets located in the cytoplasm near the cell membrane. In addition, perineural invasion was observed in the cholangiocarcinoma tissues at a positive rate of 91.7% (55/60; Fig. 1c, d).

**Fig. 1:** **a** Normal biliary duct gland tissues had regular shapes (arrow; ×200). **b** Gland tissues of in the cholangiocarcinoma patients were enlarged and disordered (arrow; ×200). **c** and **d** Intermediate cholangiocarcinoma invasion of nerve fibers (arrows; **c**: ×200 and **d**: ×400). **e** Cholangiocarcinoma patient survival is related to M3-mAChR expression. **f** Survival times of patients with cholangiocarcinoma with or without perineural invasion. Scale bars, 200 μm

Notably, M3-mAChR expression appears to be significantly correlated with the level of differentiation (*P* < 0.05), with the positive rate of M3-mAChR expression in III–IV staged tumors being higher than that in I–II staged tumors (*P* < 0.01). Similarly, expression was also correlated with lymphatic metastasis (*P* < 0.05), being higher in histopathological sections of cholangiocarcinoma with lymph node metastasis (*P* < 0.01). We also found that M3-mAChR expression is significantly associated with perineural invasion (*P* < 0.01; Table 1). The survival time of cholangiocarcinoma patients with high M3-mAChR expression was also distinctly shorter than that of patients with low M3-mAChR expression. Moreover, the survival time of cholangiocarcinoma patients was shorter when perineural invasion had occurred than in patients without perineural invasion (Fig. 1e, f). There were no connections between M3-mAChR expression and patient age, sex, tumor location (*P* ˃ 0.05). Collectively, these results show that M3-mAChR plays an important role in the invasion and metastasis of cholangiocarcinoma and affects treatment and prognosis.

**Table 1:** Clinicopathological features of patients with cholangiocarcinoma and correlations with M3 expression

Factor	n	M3 expression					*P* value
		(−)	( + )	( ++)	( +++)	Positive rate (%)	
Sex							
Male	43	5	6	14	18	88.89	0.500
Female	17	1	6	4	6	93.33	
Age							
< 59	23	2	5	7	9	91.30	0.962
≥ 59	37	4	7	11	15	89.19	
Differentiation of tumors							
High	18	3	4	5	6	83.33	0.308
Middle and poorly	42	3	8	13	18	92.86	
Lymph node metastasis							
Yes	46	1	8	15	22	97.83	0.001
No	14	5	4	3	2	64.29	
TNM stage							
I–II	16	5	5	3	3	68.75	0.002
III–IV	44	1	7	15	21	97.73	
Tumor location							
Hilar	19	2	3	6	6	88.23	0.756
Middle and distal	41	4	9	12	18	90.70	
Perineural invasion							
Yes	53	3	10	16	24	94.34	0.007
No	7	3	2	2	0	57.14	

Correlations were estimated by Fisher’s exact test. Significant when p < 0.05

### M3-mAChR mediate migration in cultured cholangiocarcinoma cells

Preliminary studies showed that both FRH0201 and RBE cells express M3-mAChR, although expression was higher in RBE cells than in FRH0201 cells (Fig. 2a, b). Notably, in RBE and FRH0201 cells treated with the M3-mAChR agonist pilocarpine, we observed an increase in the quantity of migrating cells compared with that of the untreated control group (Fig. 2c, d), suggesting that the M3-mAChR agonist significantly promoted the invasive characteristics of the cholangiocarcinoma cells. Moreover, while there was no difference between cells treated with the M3-mAChR antagonist atropine and control cells, when cells were treated with both pilocarpine and atropine, the quantity of migrating cells was reduced (Fig. 2b, c). These data suggest that the invasive capacity of the cholangiocarcinoma cells was decreased owing to antagonism of the pilocarpine-treated cells by atropine.

**Fig. 2:** Treatment with M3-mAChR agonist and antagonist alters migration in cultured cholangiocarcinoma cells. **a**, **b** Expression of M3-mAChR in FRH0201 and RBE cells. **c** Quantity of invasive RBE cells after treatment with pilocarpine (agonist) and/or atropine (antagonist). **d** Quantity of invading FRH0201 cells after treatment with pilocarpine and/or atropine

To further understand the role of M3-mAChR in cholangiocarcinoma cells, we transfected RBE cells with lentiviral vectors carrying shM3 to downregulate M3-mAChR expression (Fig. 3a). Our results show that M3-mAChR expression was downregulated in shM3-treated RBE cells, and the number of migrating cells was reduced. Furthermore, treatment with pilocarpine increased the invasive capacity of the shM3-treated RBE cells (Fig. 3b). In contrast, in FRH0201 cells, M3-mAChR expression was increased by transfecting the cells with an M3-mAChR plasmid, and this overexpression mediated an increase in cholangiocarcinoma cell invasion (Fig. 3b). Moreover, downregulation of M3-mAChR expression largely blocked invasion.

**Fig. 3:** M3-mAChR expression alters migration in cultured cholangiocarcinoma cells. **a** Lentiviral-transfected RBE cells were observed under a fluorescence microscope after viral transfection of shM3. Scale bar, 50 μm. **b** Influence of M3-mAChR expression on cholangiocarcinoma cell migration

### Perineural invasion is regulated by M3-mAChR

To investigate the role of M3-mAChR in perineural invasion of cholangiocarcinoma cells, we used an ex vivo DRG model. When the DRG from newborn Kunming mice were cultured alone (Fig. 4a-1–3), the Nissl bodies became granular after being dyed, showing obvious staining around the perinuclear region, but little staining around the edges of the nucleus (Fig. 4a–7). After Gomori staining and neurofilament protein immunohistochemical staining (NF IHC), neuritis was observed growing up from the DRG periphery, most of which showed branching and were generally present in a radial arrangement (Fig. 4a-6). Notably, when the DRG was co-cultured with untreated RBE cells, the cells appear to invade the DRG and the surrounding nerve fibers (Fig. 4b). Furthermore, when pilocarpine was added to the co-cultures, the quantity of RBE cells invading the DRG and surrounding nerve fibers was increased, suggesting that pilocarpine promotes perineural invasion during cholangiocarcinoma. The effects of pilocarpine were decreased by co-treatment with atropine, which decreased the number of RBE cells invading the DRG (Fig. 4b). Notably, atropine alone did not significantly affect the level of perineural invasion compared with that in the control group, which is consistent with our earlier cell culture data.

**Fig. 4:** M3-mAChR alters perineural invasion in cultured cholangiocarcinoma cells. **a** Growth status, survival conditions, cell size, and axon growth of dorsal root ganglion (DRG) after ex vivo culture for 36 h. **a-1** DRG anatomy. **a-2** and **a-3** Representative images showing DRG survival and growth (arrow; panel 2: ×20 and panel 3: ×40). **a-4** and **a-5** Representative images of Gomori-stained DRGs (arrow) highlighting the reticular fibers (light green) (panel 4: ×20) and neuritis occurring at the periphery (arrow; panel 5: ×40). **a-6** Representative images of NF IHC-stained DRGs highlighting the branched and radial arrangement of the neuritis structures (arrow; ×40). **a-7** Representative images of Niss1-stained DRGs showing the neuritis growing from the DRG periphery (arrow; ×40). **b** RBE cell invasion during co-culture with DRGs in the presence of different factors (arrow). The data are presented as the mean ± SD. *P < 0.05, **P < 0.01. **c** Influence of M3-mAChR expression on perineural invasion by cholangiocarcinoma cells. Scale bar, 50 μm

Furthermore, when the DRG were co-cultured with shM3-treated RBE cells, we found that although the shM3-treated RBE cells still invade the DRG, the quantity of invading cells was reduced compared with that in the untreated RBE group. Treating these DRG-shM3-RBE co-cultured cells with pilocarpine, the number of invading cells was increased (Fig. 4c). Conversely, when FRH0201 cells overexpressing M3-mAChR were co-cultured with DRG, the number of cells invading the DRG increased compared with that in the untreated FRH0201 group. Treatment these DRG-M3-FRH0201 co-cultured cells with pilocarpine, the number of invading cells was further increased (Fig. 4c). These results show that M3-mAChR expression in cholangiocarcinoma cells regulate perineural invasion.

### M3-mAChR participate in AKT-mediated EMT in cholangiocarcinoma

Through this experiment we found that pilocarpine can induce the increase of M3-mAChR protein levels in cholangiocarcinoma, and atropine blocked these changes. So we believe that pilocarpine interacts with M3-mAChR and acts through M3-mAChR.

As EMT plays a key role in cholangiocarcinoma metastasis, we examined the effects of M3-mAChR agonist and antagonist treatment on the expression of EMT factors related to the PI3K/AKT pathway in RBE cells. Our results showed that pilocarpine treatment decreases the expression of PTEN and the epithelial cell marker E-cadherin, but increases the expression AKT and the Leydig cell marker vimentin. The expression of Snail, which induces EMT, was also increased. Notably, atropine blocked these changes (Fig. 5a, b). Similarly, shM3-mediated disruption of receptor expression in the RBE cells also resulted in increased expression of PTEN and E-cadherin and decreased expression of AKT, vimentin, and Snail. In contrast, upregulation of M3-mAChR in FRH0201 cells decreased PTEN and E-cadherin expression and increased AKT, vimentin, and Snail expression (Fig. 5c, d).

**Fig. 5:** M3-mAChR agonist and antagonist influence cholangiocarcinoma cell EMT through the PTEN/AKT pathway. **a**–**d** Western blots showing the expression of the indicated EMT markers. The quantitated data are presented as the mean ± SD. *P < 0.05, **P < 0.01

To better understand the role of M3-mAChR in AKT-mediated EMT, we knocked down AKT expression in FRH0201 cells overexpressing M3-mAChR. This disruption resulted in the downregulation of M3-mAChR, Snail, and vimentin expression, whereas the expression of PTEN and E-cadherin was upregulated (Fig. 6). Moreover, when AKT was downregulated, the levels of invasion and perineural invasion were significantly decreased. We also found that down-regulating the expression of AKT can reduce the activity of MMP in cholangiocarcinoma cells. Taken together, these results showed that the AKT pathway plays a significant role in M3-mAChR-mediated invasion and perineural invasion in cholangiocarcinoma.

**Fig. 6:** M3-mAChR participate in AKT-mediated EMT in cholangiocarcinoma. **a** Western blots showing the expression of the indicated EMT markers. **b** Influence of AKT knock-down on the invasiveness of FRH0201-M3 cells. **c** Influence of AKT knock-down on the perineural invasion of FRH0201 cells. **d** Influence of AKT knock-down on MMP activity. The quantitated data are presented as the mean ± SD. *P < 0.05, **P < 0.01

## Discussion

As an important digestive organ, the biliary system is responsible for biliary secretion and excretion and is surrounded by vagus nerves that can affect and be affected by processes occurring in the biliary cells. Notably, acetyl choline acts is the main neurotransmitter in this system, and acetyl choline receptors, including nicotinic acetylcholine receptors and mAchRs, play an important functional role during signaling. mAChRs are G protein-coupled receptors that regulate adenylate cyclase, ion channels, and phosphatidylinositol lipid turnover, thus modulating various biological reactions [18, 19].

Studies have shown that the M3-mAChR is widely expressed in digestive tract tumors and may play an important role in the proliferation, differentiation, and progression of cancer [13, 14, 20–22]. Our results show that the M3-mAChR is highly expressed in cholangiocarcinoma and is closely related to the differentiation and clinical stages of the tumor as well as the presence of lymphatic metastasis. Indeed, poor cholangiocarcinoma differentiation was associated with high M3-mAChR expression. In III-IV cancers, the positive rate of M3-mAChR expression in cholangiocarcinoma was notably higher than that observed in I–II cancers, and the expression of M3-mAChR in cholangiocarcinoma patients with concomitant lymphatic metastasis was also increased. Thus, the pattern and correlation of M3-mAChR expression with survival indicate an important function for this receptor in the occurrence and development of cholangiocarcinoma along with patient prognosis.

In 1998, Wessler et al. [23] proposed the concept of the non-neuronal acetylnergic system, which is based on the non-neuronal acetylcholine system, and includes its synthetase, transporter, inactivation enzyme, and functional receptors. Functional abnormalities in this non-neuronal acetylnergic system have been related to various diseases, including inflammation, atherosclerosis, local and systemic infection, and cancer [24]. Many recent studies have also examined the interactions between neurotransmitters and tumors, particularly tumors exhibiting perineural invasion, such as cholangiocarcinoma [25–27]. In fact, abnormal neurotransmitter expression and/or receptor signaling in tumors greatly affects tumor proliferation, differentiation, and metastasis, with receptor agonists increasing these characteristics and receptor antagonists blocking them [28, 29]. In a previous study, we found that the M3-mAChR agonist pilocarpine promoted the proliferation of cholangiocarcinoma cells, increased M3-mAChR expression in cholangiocarcinoma, and enhanced the effects of M3-mAChR; all of which were blocked by treatment with the antagonist atropine [12]. In the present study, we not only verified these changes, but we also found that M3-mAChR regulate the migration and metastasis of cholangiocarcinoma cells. Our data show that when M3-mAChR expression is downregulated via receptor knock-down, the migratory capacity of the affected cholangiocarcinoma cells was low. However, when treated with the M3-mAChR agonist pilocarpine, migration was increased. A similar effect was also observed when M3-mAChR was overexpressed in cholangiocarcinoma cells. However, it appears that these enhanced effects can be blocked using atropine, highlighting the potential use of this or other antagonists in clinical treatment.

Cholangiocarcinoma is one of the deadliest malignant tumors because of the high levels of local invasion and metastasis and the insensitivity of the cells to radiotherapy and chemotherapy. The early occurrence of perineural invasion and metastasis in cholangiocarcinoma has also been shown to affect mortality rate [30]. In addition to its role in migration, we also found that high M3-mAChR expression (via overexpression) promotes perineural invasion, whereas low M3-mAChR expression (via receptor knock-down) was associated with lower levels of perineural invasion. Similar results were also observed using pilocarpine and atropine. These findings suggest that decreasing M3-mAChR expression via knock-down or antagonist treatment may limit perineural invasion of cholangiocarcinoma tumors in the clinical setting.

To understand how M3-mAChR regulate migration, perineural invasion, and metastasis in cholangiocarcinoma, we evaluated the expression and function of various factors and signaling pathways. EMT is widely known to play an essential role in metastasis and confers noninvasive cells with invasive and aggressive features [7], leading to the occurrence and progression of epithelial cell tumors [17]. The phosphatidylinositol-3-kinase (PI3K)/Akt signaling pathway plays an important role in regulating cell proliferation and EMT of malignant cells [31–33]. Our results show that downregulation of M3-mAChR expression in cholangiocarcinoma cells also decreases the expression of PTEN and the epithelial cell marker E-cadherin, while increasing that of AKT and the Leydig cell marker vimentin. These results demonstrate that downregulation of M3-mAChR blocks EMT, whereas upregulation of M3-mAChR transforms cholangiocarcinoma cells into Leydig cells, leading to invasion and metastasis. Additionally, the expression of Snail, an important factor promoting EMT, was also increased after M3-mAChR downregulation, which could subsequently activate other deviant signaling pathways.

The serine/threonine kinase AKT (also known as protein kinase B), which contains a panel of three isoforms (AKT1, AKT2 and AKT3) in mammals, is a key communicator of PI3 K signaling. Further, knockdown of AKT in FRH0201 cells overexpressing M3-mAChR which resulted in the downregulation of M3-mAChR, Snail, and vimentin expression, whereas the expression of PTEN and E-cadherin was upregulated. AKT may have negative feedback in the regulation of M3-mAChR. Moreover, when AKT was downregulated, the levels of invasion and perineural invasion were significantly decreased. We also found that down-regulating the expression of AKT can reduce the activity of MMP in cholangiocarcinoma cells which may be the cause of the decline in invasiveness. The AKT pathway appears to play a particularly prominent role in M3-mAChR signaling as downregulation of this factor significantly decreased migration, metastasis, and perineural invasion.

## Conclusions

In this study, we evaluated the changes in M3-mAChR expression in human tissue samples and in cultured tumor cells in addition to investigating the effects of these changes on migration/metastasis, perineural invasion, and EMT in cholangiocarcinoma. Our results demonstrate that M3-mAChR regulate EMT through the AKT pathway and subsequently affect perineural invasion and metastasis during cholangiocarcinoma pathogenesis. While additional work, particularly the validation of these findings in animal models of the disease, is required, this study is the first to indicate a distinct role for M3-mAChR-mediated regulation in multiple aspects of cholangiocarcinoma. Furthermore, our data also highlight a theoretical basis for blocking perineural invasion and metastasis during cholangiocarcinoma using antagonists. Taken together, this study provides essential insight into the mechanisms and potential treatment options of cholangiocarcinoma.

## Abbreviations

M3 mAchRs: M3 muscarinic acetylcholine receptors
EMT: epithelial–mesenchymal transition
PNI: perineural invasion
PTEN: phosphatase and tensin homolog
AKT: protein kinase B
shRNA: small hairpin RNA
DRG: dorsal root ganglio
PILO: pilocarpine
ATR: atropine
PI3K: phosphatidylinositol-3-kinase
